# Selected Liver Markers in Predicting the Severity of Organophosphate and Carbamate Poisoning

**DOI:** 10.1155/2022/7826396

**Published:** 2022-06-17

**Authors:** R. Senarathne, U. Hettiaratchi, L. Athiththan, H. Peiris, C. Sarathchandra, H. Senanayake, P. Weerawansa, S. Siribaddana

**Affiliations:** ^1^Department of Biochemistry, Faculty of Medical Sciences, University of Sri Jayewardenepura, Nugegoda, Sri Lanka; ^2^Department of Medicine, Faculty of Medicine and Allied Sciences, Rajarata University of Sri Lanka, Anuradhapura, Sri Lanka

## Abstract

**Background:**

Intentional ingestion of organophosphate (OP) and carbamate is a significant health issue worldwide. It causes adverse health effects on the liver. This study aimed to determine liver transaminases (AST and ALT) and bilirubin levels to assess the severity of poisoning in patients with acute OP and carbamate poisoning.

**Methods:**

A descriptive cross-sectional study was conducted on patients admitted to a selected hospital in Sri Lanka with acute OP and carbamate poisoning. The severity of poisoning was measured by RBC cholinesterase and Peradeniya Organophosphorus Poisoning scale (POP), where six clinical features were assessed based on a 3-point scale. A score of 0–3 was considered mild, 4–7 to be moderate, and 8–11 to be severe poisoning. Liver parameters such as AST, ALT, and total and direct bilirubin were measured.

**Results:**

Among the 188 screened patients, 166 were recruited. Majority were males (112, 67.5%). Kruskal–Wallis test showed significant differences in AST and ALT on admission and AST on discharge, across POP groups ((*χ*^2^ (2, *n* = 166) = 26.48, *p* ≤ 0.001), (*χ*^2^ (2, *n* = 166) = 14.31, *p*=0.001), and (*χ*^2^ (2, *n* = 157) = 11.34, *p*=0.003), respectively)). Mann–Whitney *U* test showed significantly higher AST and ALT in the moderate POP group compared to the mild POP group (AST: *U* = 1709, *z* = −4.50, *p* ≤ 0.001, *r* = 0.36; ALT: *U* = 2114, *z* = −3.04, *p*=0.002, *r* = 0.26) on admission. In addition, the treatment outcomes (duration of hospital stay and duration of ventilator assistance) were significantly correlated (*p* ≤ 0.001) with the severity of poisoning and serum AST and ALT at the time of admission.

**Conclusion:**

AST and ALT levels on admission and AST level at discharge showed significant correlations with the severity of poisoning. Treatment outcomes significantly correlated with the severity of poisoning and serum AST and ALT levels.

## 1. Introduction

Pesticide self-poisoning is one of the most common means of suicide [1]. Organophosphate (OP) compounds are cholinesterase-inhibiting chemicals that are extensively used as insecticides in agriculture due to their low cost and availability, mainly in developing countries. Self-poisoning, with OP, is estimated to kill around 200,000 people each year, mainly in the Asia Pacific region with a mortality rate between 10 and 20% [2]. The estimated number of deaths due to deliberate self-harm is 500,000 per year in rural Asia, where 60% of them are due to pesticide poisoning [3]. Sri Lanka had one of the highest rates of suicides in the world with almost 47 deaths per 100,000 individuals in 1995 [4]. There was a 50% reduction in pesticide-related suicide rate after banning some OP pesticides (dimethoate and fenthion) and paraquat (a dipyridyl herbicide) between 2008 and 2011 [5].

Evidence suggests that OP poisoning has become a major toxicological threat to humans and animals through various toxic effects such as neurotoxicity, endocrine toxicity, reproductive toxicity, immunotoxicity, and disruption of glucose homeostasis. The primary mechanism of action by OP and carbamate insecticides is the inhibition of acetylcholinesterase (AchE), an enzyme that catalyzes the hydrolysis of the neurotransmitter acetylcholine [6, 7]. In addition to cholinergic outcomes due to OP and carbamate poisoning, harmful effects on the liver have been observed in acute ingestions and chronic exposures. The underlying mechanisms are not clear, but disturbances in the antioxidant defense system, oxidative stress, apoptosis, and mitochondrial and microsomal metabolism have been suggested [8]. The toxicity of OP compounds is mediated by the generation of free radicals, which may alter the liver metabolism and is evidenced by changes in the liver enzymes [9]. Apart from a few case reports, few studies have been conducted up to date to evaluate the effect of OP compounds on the hepatobiliary system [8]. Though carbamate usage has increased, studies on carbamate poisoning and its impact on liver transaminases and bilirubin are minimal except for few animal studies. A study performed by inducing rats with carbamates had observed a significant elevation in aspartate aminotransaminase (AST) and alanine aminotransaminase (ALT) [10]. Many studies have shown increased liver transaminases in chronic exposure to OP, but few publications are available on severity and liver enzymes in acute poisoning [11].

Therefore, the present study was conducted to explore the role of AST, ALT, and bilirubin in assessing the severity of acute organophosphate and carbamate poisoning. Analysis of cholinesterase levels in RBC or plasma or analysis of OP metabolites are expensive, and facilities are not widely available in Sri Lanka, where the poisoning occurs commonly. Hence, finding a correlation between liver enzymes and the severity of OP and carbamate poisoning would benefit the treatment process in these patients.

Anuradhapura is the largest district of Sri Lanka, and agriculture is the primary employment. The paddy production statistics in 2019 and 2020 indicated the largest harvest from the Anuradhapura district. In 2014, out of the total population of 866,000 in the district of Anuradhapura, 713,919 were from families involved in agriculture. Hence, a large number are exposed to pesticides directly or indirectly. Teaching Hospital Anuradhapura (THA) is the only tertiary care hospital in the Anuradhapura district where a majority of the severe OP and carbamate-poisoned patients are treated by direct admission or transfer from other smaller hospitals in the district [12, 13]. Hence, THA was selected as the study setting for this research.

## 2. Methods

This is a descriptive cross-sectional study carried out at THA. This study assessed 188 patients over 18 years old who self-ingested OP or carbamate from August 2018 to February 2020 and were admitted to the THA. Inclusion criteria were as follows: age between 18 and 60 years, diagnosed with OP or carbamate poisoning by the clinician, patients presented with a history of OP/carbamate poisoning (poison material/bottle/label) without any prior treatment, and patients who were admitted within 24 hours of ingestion [14]. Poisoning with toxic substances other than OP and carbamate, pregnant women, ingesting poison along with alcohol, chronic drug intake, and evidence of chronic diseases (liver, renal, pancreas, malignancies, etc.) were excluded from the study.

Data were collected using an interviewer-administered questionnaire from either the guardian or the patient if possible. During the admission, sociodemographic data, poisoning history, symptoms, and medical information were recorded. Ethical approval was obtained from the ethics review committee, Faculty of Medical Sciences, University of Sri Jayewardenepura (82/17), and the ethics review committee of Rajarata University of Sri Lanka (2018/11). Proxy consent (verbal consent obtained from the person who bought the patient to the hospital, usually a parent, child, spouse, or sibling) was obtained on admission when the patient was unconscious and severely ill. Written informed consent was taken after the patient is conscious.

Severity was measured by two methods: the Peradeniya Organophosphorus Poisoning scale (POP) and red blood cell (RBC) cholinesterase level. Six common clinical features—pupil size, respiratory rate, heart rate, fasciculation, level of consciousness, and seizures—were given scores to assess severity. Each clinical feature was assessed based on a 3-point scale which varied from 0 to 2, and the details are shown in Table 1. Accordingly, a score of 0–3 was considered mild, 4–7 to be moderate, and 8–11 to be severe poisoning [15]. Since the primary mechanism of toxicity due to OP and carbamate is similar, the severity of poisoning by acute carbamate ingestion also was graded according to the POP scale (Table 1). RBC cholinesterase was measured using an assay kit based on the Ellman method when the patient was admitted to the hospital and before commencing any treatment [3, 12]. The outcome of the patient was assessed by the number of days in the hospital, death, and the requirement for ventilator-assisted breathing. Patients with respiratory failure underwent endotracheal intubation as noninvasive ventilation was not used in OP and carbamate poisoning. Patients who were ventilated or dead were considered seriously ill and others as nonseriously ill.

Aspartate transaminase (AST), alanine transaminase (ALT), direct bilirubin (D Bil), and total bilirubin (T Bil) were analyzed on admission and at discharge. Analysis was performed using the Konelab 20XT clinical chemistry autoanalyzer following the protocols given by the BIOLABO reagent kits.

Data were analyzed using SPSS version 21. Nonparametric tests were used as normal distribution was not assumed, and there were only 11 patients in one cell. Kruskal–Wallis *H* test was applied to compare liver transaminases and bilirubin among 3 POP groups (mild, moderate, and severe). Mann–Whitney *U* test was used to determine differences between each group with Bonferroni adjustments, and the effect size was calculated. Spearman's Rho test was used to examine correlations between liver transaminases (AST and ALT) with the severity of poisoning (RBC cholinesterase and POP scale) on admission and treatment outcomes (duration of hospital stay and duration of ventilator assistance).

## 3. Results

### 3.1. Baseline Data of Recruited OP and Carbamate-Poisoned Patients

After admission, 13 patients died due to OP and carbamate poisoning in the hospital giving a case fatality rate of 6.9% (13/188). Thus, we recruited 166 patients for the study, where most of them were males (112, 68%) and 49% were below 30 years. Patient recruitment details are given in Figure 1. The average hospital stay was 4 (SD ± 3) days. There were 48 seriously ill patients, 47 (28.3%) were ventilated (36 were managed in the ICU, and others were ventilated in the high-density units in the ward because of the nonavailability of ICU beds), and nine died, including one nonventilated patient, who was 26 years old, and the intermediate syndrome was the cause of death at the postmortem.

A majority of the patients (101(61%)) ingested carbamate. The mean age of male patients was 36 (SD ± 13) years, and in female patients, it was 30 (SD ± 11) years. The average volume of pesticide ingested was 58.5 (SD ± 33.5) mL, and the mean time taken for hospital admission after ingestion of poison was 82.2 (SD ± 78.7) minutes. Patients were classified into mild (87), moderate (68), and severe (11) groups according to the POP scale.

The median (interquartile range) RBC cholinesterase of AST, ALT, D Bil, and T Bil on admission were 11.6 (IQR (inter quartile range): 22.6–1.3) U/g Hgb, 39.9 (IQR: 56.75–29.47) IU/L, 19.7 (IQR: 28.97–13.8) IU/L, 0.13 (IQR: 0.19–0.13) mg/dL, and 0.55 (IQR: 0.85–0.55) mg/dL, respectively, and at discharge were 34.7 (IQR: 54.0–27.4) IU/L, 21.3 (IQR: 29.0–13.85) IU/L, 0.14 (IQR: 0.19–0.10) mg/dL, and 0.56 (IQR: 0.82–0.39) mg/dL. AST was higher compared to ALT in most patients. Higher AST compared to ALT was observed in 92% of mild poisoned group, 91% of moderate poisoned group, and all patients in the severe poisoned group (defined according to the POP scale).

RBC cholinesterase on admission declined, while AST and ALT on admission elevated with increased severity of poisoning categorized by the POP scale (Table 2). Though significant median differences in RBC cholinesterase, AST, and ALT were observed between mild-moderate and mild-severe groups according to the POP scales, we could not detect a significant median difference in RBC cholinesterase and liver transaminases between moderate and severe.

Poisoned groups (Table 3): bilirubin levels did not show any significant differences across the POP groups (Table 2).

However, there is a significant difference in patient-related outcomes (duration of hospital stay and number being ventilated) among all three groups (Table 3).

Among the seriously ill patients (patients who were ventilated or dead), 32 (66.7%) were males. Of the other patients, 80 (67.8%) were males (*p*=0.51). The mean age (SD) of seriously ill patients (38 ± 14 years) was significantly higher (*p*=0.030) compared to nonseverely ill patients (33 ± 13 years). The proportion of patients who have ingested carbamate was not statistically significant (*p* value = 0.12) between seriously ill patients (3 (68.7%)) and not seriously ill patients (68 (57.6%)). Significantly higher (*p* ≤ 0.001) volume of poison was ingested by the seriously ill patients (83.1 ± 33.9 mL) compared to the other patients (48.5 ± 27.8 mL). On admission, RBC cholinesterase level and liver transaminases were significantly elevated in seriously ill patients (Table 4).

According to both severity assessment methods of poisoning (RBC cholinesterase and POP scale), liver transaminases on admission significantly correlated with the severity of poisoning. There were no correlations detected between bilirubin (D Bil and T Bil) and the severity of poisoning. Patient outcomes (duration of hospital stay and number of patients on ventilator) significantly correlated with transaminases level on admission (Table 5).

On further analysis, 16 patients (9.6%) and one patient (0.6%) had AST and ALT elevated more than three times normal and six patients (3.6%) had AST elevated more than five times normal. Two patients had T Bil more than 2.5 mg/dL. However, 153 (92.2%) had AST levels higher than ALT.

## 4. Discussion

The poisoning by pesticides that inhibit cholinesterase (OP and carbamate) is a major health burden [16]. Our findings confirm a positive correlation of liver transaminases with the duration of the hospital stays, the severity of poisoning measured by RBC cholinesterase, a POP scale developed objectively to assess the severity of poisoning based on physical signs, and the need for respiratory support. The correlation obtained between transaminases and patient outcome demonstrate the potential of analyzing liver enzymes as a marker of severity. Though the studies related to acute OP poisoning are limited, studies conducted on (both humans and animals) long-term exposure to OP have observed a significant elevation in liver enzymes [17, 18].

A single-center study in Nepal has observed a significant correlation between AST and severity of poisoning based on the serum cholinesterase level. However, ALT, D Bil, and T Bil did not show any significant association with the severity of poisoning [19]. In a Turkish study, both AST and ALT levels were high among patients poisoned with OP [20]. Studies related to OP and carbamate poisoning have not observed statistically significant differences in the values of T Bil and D Bil, confirming the finding of the current study [19, 20]. We assessed liver transaminases and bilirubin both on admission and at discharge and found to have a significant correlation between AST with the severity of poisoning for both admission and discharge, while all the other studies have focused on liver enzymes at a single time point during the hospital stay [19–21]. The underlying mechanism for the elevation of liver transaminases is not clear, but disturbances in the antioxidant defense system, oxidative stress, apoptosis, and mitochondrial and microsomal metabolism have been suggested [8].

Although the rise of liver transaminases was not pronounced, with only 4% having AST more than five times normal, the modest and subtle increases may have to be considered [22]. Another study has also shown elevated AST in a majority of the patients with decreased serum cholinesterase levels compared to ALT [20]. The other significant finding in this study is that the elevation of the AST/ALT ratio is more than 90% of patients. AST has cytosolic and mitochondrial isoenzymes and is found in the heart, kidney, brain, skeletal muscle, and red blood cells. ALT is a cytosolic enzyme mainly found in the liver [23]. Hence, elevation of AST can be attributed to the pathology outside the liver. Also, with the high background prevalence of NAFLD (32.6% in urban areas in Sri Lanka), interpreting a mild increase in liver enzymes is a challenge [24].

Determination of RBC cholinesterase level in blood is considered an accurate and fastest method of assessing the severity of anticholinesterase pesticide poisoning [3, 25]. However, it is not widely available. Hence, the POP, a severity scale based on physical signs, had been developed to assess the severity of OP poisoning [15]. Though significant median differences in RBC cholinesterase, AST and ALT were observed between mild and moderate groups according to the POP scale, we could not detect significant median differences in RBC cholinesterase and liver transaminases between moderate and severe poisoning groups based on the severity of POP scale. But the duration of hospital stays and the number of patients ventilated differed significantly between the moderate and severe groups of POP. These two (duration of hospital stays and the number of patients ventilated) patient-related outcomes indicate the difference between the three groups. However, 50% of patients in the moderate POP group needed ventilation and were misclassified.

The death rate (6.9%) of the present study was minimal compared to other developing countries. This may be attributed to the better health care service in Sri Lanka, less time elapsed between hospital admission and ingestion, or the quantity (little amount) ingested [26, 27].

In the present study, OP and carbamate poisoning were more common among males. Several other studies have reported a male predominance in acute pesticide intoxication [25, 28]. Almost half of the patients (49%) were less than 30 years in our study. Others have also confirmed that younger people are more vulnerable to self-poisoning [28].

The drawback of this study was assessing the severity with the POP scale, which depends on the observations recorded by the clinician in the hospital notes. Some variables in the POP scale (e.g., fasciculation) were not regularly recorded. Often, the clinician is a first-year doctor who is fresh from a medical school. In addition, time taken to reach the hospital and volume ingested were obtained through a questionnaire from the intimate member accompanying the patient, and bias reporting is a possibility. Sample collection of this study was limited to a single study setting as an expansion to other sites was not feasible. The other drawback is the measurement of RBC cholinesterase by the Ellman method. This has been criticized for several reasons [29].

## 5. Conclusion

AST and ALT level on admission and AST level at discharge showed significant correlations with the severity of poisoning. Treatment outcomes significantly correlated with the severity of poisoning as well as serum AST and ALT levels.

However, using transaminases or derived values as a proxy indicator for assessing the severity of poisoning needs further consideration.

## Figures and Tables

**Figure 1:** Details of patient recruitment.

**Table 1:** Peradeniya Organophosphate Poisoning scale.

Parameter	Criteria	Score
Pupil size	≥2 mm	0
	<2 mm	1
	Pinpoint	2

Respiratory rate	<20/min	0
	≥20/min	1
	≥20/min with central cyanosis	2

Heart rate	>60/min	0
	41–60/min	1
	<40/min	2

Fasciculation	None	0
	Present, generalized/continuous	1
	Both generalized and continuous	2

Level of consciousness	Conscious and rationale	0
	Impaired response to verbal command	1
	No response to verbal command	2

Seizures	Absent	0
	Present	1

0–3: mild poisoning; 4–7: moderate poisoning; 8–11: severe poisoning.

**Table 2:** Comparison of RBC cholinesterase, liver transaminases, and bilirubin and severity on admission and at discharge among the POP groups.

Biochemical test	Mild POP median (IQR)	Moderate POP median (IQR)	Severe POP median (IQR)	*X* ^2^ (*P* value)
On admission^^^ (*n* = 166)	87	68	11	
RBC cholinesterase (U/g Hgb)	22.4 (9.9–25.6)	3.0 (1.0–12.0)	0.7 (0.3–2.1)	47.41 (≤0.001)^*∗*^
ALT (IU/L)	17.8 (11.9–23.2)	22.3 (15.3–39.2)	22.7 (17.3–54.7)	14.32 (≤0.001)^*∗*^
AST (IU/L)	33.9 (25.8–43.3)	47.4 (35.0–65.8)	73.2 (26.1–121.5)	26.48 (≤0.001)^*∗*^
AST/ALT	1.92 (1.49–2.70)	2.15 (1.59–2.83)	2.25 (1.06–3.37)	0.846 (0.655)
Direct bilirubin (mg/dL)	0.12 (0.10–0.18)	0.13 (0.10–0.19)	0.14 (0.80–0.24)	0.23 (0.89)
Total bilirubin (mg/dL)	0.53 (0.37–0.81)	0.56 (0.34–0.92)	0.51 (0.42–0.69)	0.52 (0.78)
Hospital stay (days)	3 (3–4)	5 (4–7)	8 (6–10)	49.51 (≤0.001)^*∗*^
No. of patients being ventilated (%)	2 (2.3)	34 (50.0)	11 (100.0)	72.18 (≤0.001)^*∗*^
No. of deaths (%)	2 (2.3)	5 (7.3)	2 (18.2)	5.60 (0.06)
Seriously ill patients (%)^∗∗^	03 (3.5)	34 (50.0)	11 (100.0)	
RBC cholinesterase (U/g Hgb)	9.4 (6.5–15.8)	2.0 (0.7–7.8)	0.8 (0.5–2.5)	4.18 (0.12)
ALT (IU/L)	17.6 (13.0–19.9)	25.7 (15.8–48.5)	30.7 (19.7–48.9)	2.50 (0.29)
AST (IU/L)	54.9 (45.2–71.9)	50.0 (35.0–87.1)	73.2 (46.2–121.5)	1.21 (0.55)
AST/ALT	4.21 (3.34–4.63)	2.08 (1.53–2.84)	2.25 (1.60–3.37)	4.14 (0.13)
Direct bilirubin (mg/dL)	0.25 (0.23–0.25)	0.14 (0.11–0.20)	0.14 (0.80–0.21)	3.44 (0.18)
Total bilirubin (mg/dL)	0.73 (0.68–0.74)	0.53 (0.35–0.87)	0.51 (0.42–0.61)	1.40 (0.50)
At discharge^#^ (*n* = 157)	85	63	09	
ALT (IU/L)	17.0 (13.4–26.7)	23.5 (14.2–32.7)	23.0 (20.7–38.4)	5.74 (0.06)
AST (IU/L)	30.0 (25.4–42.3)	37.9 (29.9–56.8)	40.1 (31.0–80.3)	11.35 (≤0.001)^*∗*^
Direct bilirubin (mg/dL)	0.14 (0.10–0.19)	0.14 (0.10–0.19)	0.10 (0.08–0.16)	3.10 (0.21)
Total bilirubin (mg/dL)	0.59 (0.40–0.90)	0.56 (0.38–0.78)	0.38 (0.31–0.53)	4.29 (0.12)

IQR = interquartile range; *X*^2^: chi-square; ^*∗*^ significant at 0.01 level; ^ included dead and seriously ill patients.^∗∗^Seriously ill patients were shown separately but included in the on-admission category, ^#^Seriously ill patients but not dead.

**Table 3:** Differences of RBC cholinesterase and liver transaminases between POP groups.

Biochemical test	Mild-moderate *Z* score (U)	*r*	Mild-severe *Z* score (U)	*r*	Moderate-severe *Z* score (U)	*r*
RBC cholinesterase	−6.23 (1228)^*∗*^	0.50	−4.05 (119)^*∗*^	0.43	−1.80 (247)	0.20
AST admission	−4.50 (1709)^*∗*^	0.36	−3.26 (189)^*∗*^	0.33	−1.69 (255)	0.19
ALT admission	−3.04 (2114)^*∗*^	0.25	−2.92 (219)^*∗*^	0.30	−1.13 (294)	0.13
AST discharge	−3.18 (1856)^*∗*^	0.26	−1.67 (252)	0.17	−0.52 (253)	0.06
Duration of hos. stay	−6.62 (1168)^*∗*^	0.50	−3.64 (168)^*∗*^	0.37	−2.18 (222)^*∗*^	0.25
No. of patients being ventilated	−6.96 (1547)^*∗*^	0.56	−8.96 (11)^*∗*^	0.91	−3.08 (187)^*∗*^	0.35

^*∗*^ *p* value is significant at 0.05/3 level; *r* = effect size; 0.1 = small effect; 0.3 = medium effect; 0.5 = large effect.

**Table 4:** Differences in RBC cholinesterase and liver transaminases between seriously ill patients (*n* = 48) and nonseriously ill patients on admission.

Biochemical test	Mann–Whitney *U*	*Z*	*P* value	*r*
RBC cholinesterase	1371.5	−5.20	≤ 0.001	0.40
AST admission	1601.5	−4.382	≤ 0.001	0.34
ALT admission	1974.5	−3.054	0.002	0.24
Direct bilirubin	2401.5	−1.536	0.125	0.12
Total bilirubin	2822.0	−0.036	0.972	0.00

^*∗*^ *p* value is significant at 0.05 level; *r* = effect size; 0.1 = small effect; 0.3 = medium effect; 0.5 = large effect. *Z* = chi-square.

**Table 5:** Correlations between biochemical and clinical parameters and the severity of poisoning measured by RBC cholinesterase and POP scale on admission.

Treatment outcomes of patient	AST on admission	ALT on admission
Duration of hospital stay	0.31^∗∗^	0.25^∗∗^
Duration of ventilator assistance	0.33^∗∗^	0.26^∗∗^
Admission RBC cholinesterase	−0.26^∗∗^	−0.17^*∗*^
Admission POP scale	0.43^∗∗^	0.27^∗∗^

^∗∗^Correlation is significant at 0.01 level. ^*∗*^Correlation is significant at 0.05 level.

## Data Availability

The datasets used to support the findings of this study are available from the corresponding author upon request.
